The article "Assessment of Three Mathematical Prediction Models for Forecasting the COVID-19 Outbreak in Iran and Turkey" was published in 2020. Journal: Comput Math Methods Med.

# Assessment of Three Mathematical Prediction Models for Forecasting the COVID-19 Outbreak in Iran and Turkey

**DOI:** 10.1155/2020/7056285

**Published:** 2020-11-21

**Authors:** Majid Niazkar, Gökçen Eryılmaz Türkkan, Hamid Reza Niazkar, Yusuf Alptekin Türkkan

**Affiliations:** ^1^Department of Civil and Environmental Engineering, Shiraz University, Shiraz, Iran; ^2^Department of Civil Engineering, Bayburt University, Bayburt, Turkey; ^3^Medical Student, Student Research Committee, Gonabad University of Medical Sciences, Gonabad, Iran; ^4^Department of Mechanical Engineering, Bayburt University, Bayburt, Turkey

## Abstract

COVID-19 pandemic has become a concern of every nation, and it is crucial to apply an estimation model with a favorably-high accuracy to provide an accurate perspective of the situation. In this study, three explicit mathematical prediction models were applied to forecast the COVID-19 outbreak in Iran and Turkey. These models include a recursive-based method, Boltzmann Function-based model and Beesham's prediction model. These models were exploited to analyze the confirmed and death cases of the first 106 and 87 days of the COVID-19 outbreak in Iran and Turkey, respectively. This application indicates that the three models fail to predict the first 10 to 20 days of data, depending on the prediction model. On the other hand, the results obtained for the rest of the data demonstrate that the three prediction models achieve high values for the determination coefficient, whereas they yielded to different average absolute relative errors. Based on the comparison, the recursive-based model performs the best, while it estimated the COVID-19 outbreak in Iran better than that of in Turkey. Impacts of applying or relaxing control measurements like curfew in Turkey and reopening the low-risk businesses in Iran were investigated through the recursive-based model. Finally, the results demonstrate the merit of the recursive-based model in analyzing various scenarios, which may provide suitable information for health politicians and public health decision-makers.

## 1. Introduction

The novel coronavirus disease (COVID-19) has become a worldwide health concern shortly after it was identified in Wuhan City of Hubei Province of China in December of 2019. COVID-19 has become a widespread infectious disease and affected many different countries worldwide. By 15 September 2020, it has affected more than 28 million people around the globe. Additionally, more than 915,000 deaths have been reported due to COVID-19 until 15 September 2020 [1]. Coronaviruses are common pathogens between vertebrates and humans, which are disreputable worldwide due to the outbreaks of the Severe Acute Respiratory Syndrome (SARS) and the Middle East Respiratory Syndrome (MERS) in 2002-2003 and 2012, respectively [1, 2]. In addition, severe acute respiratory syndrome coronavirus 2 (SARS-COV-2) is a newly recognized member of the coronaviruses family with a high rate of human-to-human transmission. Since COVID-19 is known to be simply transmitted by respiratory pathways, health politicians in affected countries have adopted various strict preventive measures, such as social distancing, travel bans, and different levels of quarantine [3]. The aforementioned applied preventive measures inevitably affected daily humans' lives. Furthermore, the COVID-19 pandemic has brought about an excessive burden on healthcare systems [4]. In this regard, providing an accurate perspective of the COVID-19 outbreak through estimation models is essential to adopt precise strategies and risk assessment analysis. Moreover, the efficacy of applied measurements, the number of facilities required such as hospital beds, mechanical ventilators, and possible effective drugs can be calculated through estimation models [3].

The article "Assessment of Three Mathematical Prediction Models for Forecasting the COVID-19 Outbreak in Iran and Turkey" was published in 2020. Journal: Comput Math Methods Med.

For this purpose, numerous prediction models have been proposed in the literature, which may be categorized into mathematical models [4–7] and soft computing approaches [3, 8, 9]. The former has many different types including simple explicit equations to a complicated system of equations with many parameters required to be calibrated. The soft computing techniques use a part of data to capture the pandemic trend, which enables them to predict an approximation of future confirmed cases [9]. Both of these two types of prediction models require data either to calibrate parameters or to train intelligence-based models. Additionally, their predictions may be accompanied by uncertainty and marginal unreliability. Such uncertainties are due to various reasons such as the unreliability of reported official data, the number of testing, and the negligence of asymptomatic carriers in reported data [3].

Among different kinds of mathematical models, simple explicit equations with a few calibrating parameters may be one of the simplest methods for predicting the COVID-19 outbreak. For instance, Li et al. [10] used an exponential function to predict the trend of COVID-19, and they predicted that the COVID-19 pandemic will end in China after March 20, 2020, and infects about 52000 to 68000 individuals and leads to about 2400 deaths [10]. This long-term prediction, which is proved to be inaccurate based on the current data, underestimated the COVID-19 outbreak. Also, Fu et al. [11] used the Boltzmann function to estimate the potential total numbers of confirmed cases in different regions of China based on the daily cumulative number of confirmed cases [11]. H. R. Niazkar and M. Niazkar [4] claimed that a second-order polynomial equation with constant coefficients is not adequate for the prediction of the COVID-19 outbreak in Thailand from 20 January to 29 February 2020. They also suggested developing a prediction model based on the confirmed cases rather than imported infected cases [4]. Fanelli and Piazza [12] found an iterative power-law relationship between the confirmed cases of two consecutive days. Based on their findings, they proposed a recursive-based model for predicting the COVID-19 outbreak, while they tested it for China, Italy, and France [12]. Moreover, Beesham [13] recommended a three-coefficient exponential model for predicting the COVID-19 in South Africa. Despite the simplicity of explicit mathematical models application, the accuracy of these COVID-19 prediction models recommended in the literature needs to be assessed. Moreover, no studies have been compared the accuracy of these suggested explicit mathematical models in a bid to determine the most accurate prediction models. Also, various interventions and preventive measures affect the trend of the COVID-19 outbreak, and such impacts should be addressed through revisiting the calibration of mathematical model parameters.

The article "Assessment of Three Mathematical Prediction Models for Forecasting the COVID-19 Outbreak in Iran and Turkey" was published in 2020. Journal: Comput Math Methods Med.

This research is aimed at assessing and comparing the accuracy of three recommended simple explicit mathematical COVID-19 prediction models with a few calibrating parameters. These models were applied to capture temporal variations of confirmed and death cases due to COVID-19 in Iran and Turkey. Such investigations may help to select a more accurate COVID-19 prediction model and provide a better perspective of the outbreak.

## 2. Materials and Methods

### 2.1. Data Source

The WHO official website has reported the outbreak data of COVID-19 each and every day since 20 January 2020 [1]. The daily confirmed cases and death data of Iran and Turkey were gathered from the WHO situation reports and the Ministry of Health in the Republic of Turkey, respectively [1, 14]. The data were divided into two parts named train data and test data. The former was utilized to calibrate parameters of mathematical prediction models, while the latter was used for comparison purposes. The data records of Iran and Turkey start from 20 February and 10 March 2020, respectively, while 14 May 2020 is the end date of the train data for both countries. Moreover, the test data are from 15 May to 4 June 2020 for Iran and Turkey. Based on the WHO reports, these two countries are among those on which the outbreak of COVID-19 has significant impacts. These data were analyzed using Excel software, which provides suitable facilities for data analysis and numerical implementation [15].

The article "Assessment of Three Mathematical Prediction Models for Forecasting the COVID-19 Outbreak in Iran and Turkey" was published in 2020. Journal: Comput Math Methods Med.

### 2.2. Mathematical Prediction Models

Various types of mathematical prediction models have been suggested for estimating the COVID-19 outbreak in the literature. Among the earliest proposed methods, three mathematical models were selected in this study because they (1) are easy to apply, (2) have explicit and relatively simple mathematical functions, (3) contain a few calibrating parameters, (4) do not need any advanced software to apply them, and (5) have shown promising results according to the preliminary studies. The performances of these three mathematical prediction models for the COVID-19 outbreak are investigated. These models are presented in the following:

### 2.3. A Recursive-Based Prediction Model

It was found that the number of confirmed cases at day *t* has a power-law relation with confirmed cases at day *t* − 1. The same relation was also observed for death and recovered cases [12]. Based on these time-lag relationships, a recursive-based prediction model was proposed to forecast the COVID-19 outbreak. According to this mathematical prediction model, the power-law relations for estimating confirmed and death cases due to COVID-19 are shown in Equation (1) to Equation (2), respectively [12]:

(1) $$\begin{array}{c} C\left(t\right)=\alpha_{1}{\left[C\left(t-1\right)\right]}^{\beta_{1}}, \end{array}$$

(2) $$\begin{array}{c} D\left(t\right)=\alpha_{2}{\left[D\left(t-1\right)\right]}^{\beta_{2}}, \end{array}$$

where *C*(*t*) and *C*(*t* − 1) are the cumulative number of confirmed cases at days *t* and *t* − 1, respectively; *α*_1_*α*_2_, *β*_1_, and *β*_2_ are fixed-value coefficients; and *D*(*t*) and *D*(*t* − 1) are total death cases at days *t* and *t* − 1, respectively.

The coefficients of Equation (1) can be determined by curve fitting of a recurrence plot, where its horizontal and vertical axes are *C*(*t* − 1) and *C*(*t*), respectively. Likewise, the plot of *D*(*t*) versus *D*(*t* − 1) can provide the coefficients of Equation (2). These curves can be plotted by available records of confirmed cases of the train data with a logarithmic scale. Therefore, in the calibration of two coefficients, the recurrence-based method enables it to be used as a prediction model for the spreading of COVID-19.

### 2.4. A Boltzmann Function-Based Prediction Model

The Boltzmann function was used to develop a prediction model for predicting the COVID-19 outbreak [11]. The derived relation, which is shown in Equation (3), is related to the sigmoid function except for a linear transform [11]:

(3) $$\begin{array}{c} C\left(t\right)=A_{2}+\frac{A_{1}-A_{2}}{1+e^{\left(t-t_{0}\right)/\Delta t}}, \end{array}$$

where *A*_1_, *A*_2_, *t*_0_, and Δ*t* are constant coefficients. To be more specific, *A*_1_ represents those infected cases that may not spread SARS-COV-2 to healthy people, while *A*_2_ denotes an estimation of potential confirmed cases of COVID-19. The four constant coefficients shown in Equation (3) need to be calibrated using the train data of each country. Additionally, a similar relation to Equation (3) can be presented for predicting death cases of the COVID-19 outbreak.

The article "Assessment of Three Mathematical Prediction Models for Forecasting the COVID-19 Outbreak in Iran and Turkey" was published in 2020. Journal: Comput Math Methods Med.

### 2.5. Beesham's Prediction Model

Since the spreading rate of the COVID-19 outbreak was increasing rapidly, several models with exponential function have been recommended for predicting the COVID-19 outbreak in the literature [13]. Likewise, Beesham's mathematical model, which was recommended for predicting the confirmed cases of the COVID-19 in South Africa [13], includes an exponential function. This prediction model is presented in Equation (4) [13]:

(4) $$\begin{array}{c} C\left(t\right)={at}^{b}e^{ct}, \end{array}$$

where *a*, *b*, and *c* are constant coefficients. These coefficients can be determined through a common regression analysis or parameter estimation process for the train data. Moreover, a similar relation of Equation (4) can be utilized for the estimation of death cases.

### 2.6. Performance Evaluation Criteria

In order to investigate and compare the performances of different mathematical prediction models, three metrics, which are written for the confirmed cases, were used [16]

(5) $$\begin{array}{c} \text{ARE}\left(t\right)=\left|\frac{C_{\text{observed}}\left(t\right)-C_{\text{estimted}}\left(t\right)}{C_{\text{observed}}\left(t\right)}\right|, \end{array}$$

(6) $$\begin{array}{c} \text{AARE}=\frac{\sum_{t=1}^{N}\text{A}\text{RE}\left(t\right)}{N}, \end{array}$$

(7) $$\begin{array}{c} R^{2}={\left(\frac{\sum_{t=1}^{N}\left[\left(C_{\text{observed}}\left(t\right)-\left(\left(\sum_{t=1}^{N}C_{\text{observed}}\left(t\right)\right)/N\right)/N\right)\left(C_{\text{estimated}}\left(t\right)-\left(\left(\sum_{t=1}^{N}C_{\text{estimated}}\left(t\right)\right)/N\right)\right)\right]}{\sqrt{\sum_{t=1}^{N}\left[{\left(C_{\text{observed}}\left(t\right)-\left(\left(\sum_{t=1}^{N}C_{\text{observed}}\left(t\right)\right)/N\right)\right)}^{2}{\left(C_{\text{estimated}}\left(t\right)-\left(\left(\sum_{t=1}^{N}C_{\text{estimated}}\left(t\right)\right)/N\right)\right)}^{2}\right]}}\right)}^{2}, \end{array}$$

where ARE(*t*) is the absolute relative error calculated at day *t*, *C*_observed_(*t*) and *C*_estimted_(*t*) are the observed and estimated number of cumulative confirmed cases at day *t*, respectively, AARE is the average absolute relative error, *N* is number of data, and *R*^2^ is determination coefficient. Based on Equations (5)–(7), the lower ARE(*t*) and AARE, the more accurate the estimations are, whereas the higher *R*^2^, the closest the predictions are to the observed values.

The article "Assessment of Three Mathematical Prediction Models for Forecasting the COVID-19 Outbreak in Iran and Turkey" was published in 2020. Journal: Comput Math Methods Med.

## 3. Results

The three mathematical prediction models were applied to forecast the confirmed and death cases due to COVID-19 in Iran and Turkey. The results achieved by each model are presented separately in the following:

### 3.1. Results of the Recursive-Based Prediction Model

As previously mentioned, the recursive-based prediction model has a power-law formula with two constant coefficients. In order to determine *α* and *β* of Equation (2), iterative one-day time-lag maps were plotted for the confirmed and death cases of the COVID-19 outbreak in Iran and Turkey. The recurrence plots of Iran and Turkey are depicted in Figure 1 for the train data. As shown, the one-day time-lag relationship of the recursive-based model was applied to the confirmed and death cases of COVID-19 in Iran and Turkey. The trend line that fits each recurrence plot shown in Figure 1 delineates values of *α* and *β*. For instance, the number of cumulative confirmed cases of COVID-19 in Iran can be estimated by implementing the values of *α* = 2.3644 and *β* = 0.9242 into Equation (1). In addition to the obtained values of *α* and *β*, Figure 1 presents the time period used in the recurrence plots.

The confirmed and death cases of COVID-19 estimated by the recursive-based model are depicted in Figure 2. It compares the observed data and the estimated values for Iran and Turkey for the train data. Moreover, the predicted values with ARE ≤ 0.1, which are considered to be acceptably accurate estimation results, are shown with different symbols than those with ARE higher than 0.1. This presentation is not only to illustrate how each prediction model performs but also to compare the estimation results. According to Figure 2, the recursive-based model estimated confirmed and death cases for the first several days with ARE higher than 0.1. This part of data has either a plateau or a slow-increasing trend, while the rest has a relatively rapidly increasing trend. The incapability of mathematical prediction models for providing acceptably accurate results due to variations of the COVID-19 outbreak (because of a plateau, a slow-increasing trend or trend changes) was observed in previous studies in the literature [3]. Based on Figure 2, it may imply that the recursive-based model performs better for Iran than Turkey for the train data. Particularly, the numbers of days with ARE ≤ 0.1 are 75 and 77 (both out of 88) days for the confirmed and death cases in Iran, respectively, while the former and latter numbers are 51 (out of 65) and 49 (out of 59) days for Turkey. Hence, the recursive-based model performs better for Iran than Turkey for the train data.

The article "Assessment of Three Mathematical Prediction Models for Forecasting the COVID-19 Outbreak in Iran and Turkey" was published in 2020. Journal: Comput Math Methods Med.

### 3.2. Results of the Boltzmann Function-Based Prediction Model

The four coefficients of the Boltzmann function-based model were calibrated using the Generalized Reduced Gradient (GRG) algorithm, which is embedded in MS Excel [15]. This first-order optimization algorithm has been successfully used for many other applications in the literature [17–19]. The calibrated coefficients were utilized to estimate the confirmed and death cases of COVID-19 in Iran and Turkey. The results estimated by the Boltzmann function-based model are compared with the observed records in Figure 3 for the train data. As shown, the values of coefficients and *R*^2^ are presented for the estimations in Figure 3. Similar to the results depicted in Figure 2, the Boltzmann function-based model estimated the confirmed and death cases with ARE > 0.1 in the first period of the data. Although ARE values for the rest of data predicted by the Boltzmann function-based model are lower than or equal to 0.1, Figure 3 shows a discrepancy between the estimated and observed values with ARE lower than 0.1, which becomes more distinct at the end of the period considered. Moreover, the numbers of days of the estimated confirmed and death cases in Iran with ARE ≤ 0.1 are 64 and 57 (both out of 85) days, respectively. The corresponding results are 44 (out of 66) and 42 (out of 59) for Turkey, respectively. These results clearly indicate that the Boltzmann function-based model achieved better estimation results than for Turkey for the train data.

### 3.3. Results of Beesham's Prediction Model

The calibration of the three coefficients of Beesham's model was conducted using the GRG algorithm.  Figure 4 presents the estimated results for the train data, the calibrated coefficients, and the corresponding *R*^2^. As shown, ARE values of the first part of data are higher than 0.1, which is similar to those of other mathematical methods considered in this study. Additionally, the numbers of days with ARE ≤ 0.1 for estimating the confirmed and death cases in Iran are 47 and 51 (both out of 85) days, while the corresponding values are 40 (out of 66) and 36 (out of 59) days for Turkey data, respectively. Based on Figure 4 and the mentioned results, Beesham's prediction model performs better for Turkey than Iran for the train data.

## 4. Discussion

Figure 5 compares the observed and estimated confirmed cases of COVID-19 in Iran and Turkey for the test data (15 May to 4 June). These data were not used in the calibration process of the mathematical prediction models. As depicted in Figure 5, the recursive-based model achieved the closest estimations to the observed confirmed cases of COVID-19 in both Iran and Turkey based on *R*^2^. Furthermore, Figure 5 indicates that the Boltzmann function-based prediction model and Beesham's prediction model underestimated the number of confirmed cases for the test data, while the discrepancy between the observed and the values predicted by these two models increase as time passes. As a result, the Boltzmann function-based prediction model and Beesham's prediction model obtained estimations with ARE ≤ 0.1 for the first part of the test data, while the second part of data was estimated with ARE > 0.1. On the contrary, the estimations carried out by the recursive-based model yielded to ARE ≤ 0.1 for the whole period of the test data.

The article "Assessment of Three Mathematical Prediction Models for Forecasting the COVID-19 Outbreak in Iran and Turkey" was published in 2020. Journal: Comput Math Methods Med.

The observed and predicted death cases due to COVID-19 in Iran and Turkey were computed for the test data and compared in Figure 6. As shown, the recursive-based model reaches to the closest estimations of COVID-19 death cases in Iran and Turkey for the test data. This result is also in agreement with *R*^2^ values presented in Figure 6. To be more specific, the best *R*^2^ value (*R*^2^ = 0.999) was obtained by the recursive-based model, whereas Beesham's prediction model yielded to the worst *R*^2^ value (*R*^2^ = 0.419) for death cases in Turkey. Based on Figures 2–6, *R*^2^ values achieved by the Boltzmann function-based prediction model and Beesham's prediction model for the test data are lower than *R*^2^ values obtained by the same models for the train data. However, the recursive-based model resulted in quite the same *R*^2^ values for both train and test data. Based on Figure 6, the recursive-based model and Beesham's prediction model forecasted the death cases with ARE ≤ 0.1 for all test data. However, the Boltzmann function-based prediction model estimated death cases with ARE ≤ 0.1 for the first half of the test data and with ARE > 0.1 for the second half of the test data. Therefore, Figures 5 and 6 demonstrate that the recursive-based model outperforms other mathematical models for predicting the confirmed and death cases of COVID-19 for the test data in Iran and Turkey.

As shown in Figures 1–4, all methods achieved acceptably high values for *R*^2^, whereas they have different performances in terms of ARE and AARE for the train data. This indicates that considering only *R*^2^ for evaluating the accuracy of a prediction model may not be technically enough and other criteria like AARE may also need to be investigated. In this regard, the performances of each mathematical prediction model considered in this study are compared in Figure 7 in terms of AARE for both train and test data. According to Figure 7, the AARE values obtained by the recursive-based model for the confirmed cases of the train data are 0.05 and 0.12 for Iran and Turkey, while AARE values for death cases are 0.03 and 0.06 in Iran and Turkey, respectively. Additionally, AARE values obtained by the Boltzmann function-based model for the confirmed cases of the train data are 16.54 and 77.41 for Iran and Turkey, respectively, which are significantly larger than those by the recursive model. Also, the Boltzmann function-based model reached 2.86 and 2.14 for AARE values of the death cases the train data in Iran and Turkey, respectively. Based on Figure 7, AARE values for the confirmed cases of Iran and Turkey are 0.47 and 0.43 for the train data, while AARE values for the death cases are 0.97 and 0.50 for Iran and Turkey, respectively. Furthermore, the estimation results of Beesham's model are also much better than those of the Boltzmann function-based model in terms of AARE for the confirmed (train and test data) and death (only train data) cases. Likewise, Figure 7 shows that the recursive-based model yielded to the lowest values of AARE for both confirmed and death cases for the test data in Iran and Turkey. Comparing the results of different models shown in Figure 7 obviously demonstrates that the recursive-based model performs the best for predicting the COVID-19 outbreak in Iran and Turkey in terms of AARE.

The article "Assessment of Three Mathematical Prediction Models for Forecasting the COVID-19 Outbreak in Iran and Turkey" was published in 2020. Journal: Comput Math Methods Med.

One of the important characteristics of a prediction model is how accurate it estimates the peak of an outbreak. For this purpose, the performances of the three mathematical prediction models for forecasting the peak confirmed and death cases of COVID-19 in the train data were compared in Table 1. As shown, the recursive-based model achieved the lowest ARE for predicting the peak of the confirmed cases in both Iran and Turkey, while the best ARE for estimating the peak of COID-19 death cases was obtained by the Boltzmann function-based model for Iran and Turkey. In Table 1, all the estimated values, except the death cases predicted by the Boltzmann function-based model for Turkey, are lower than the corresponding observed values. This indicates that the three mathematical prediction models underestimated almost all peak values of COVID-19 confirmed and death cases that occurred in Iran and Turkey.

Since the recursive-based prediction model was found to perform the best among the three mathematical prediction models considered in this study, it was used to investigate how preventive measurements may not only be implemented into the mathematical prediction model but also have impacts on estimations. Generally, applying effective interventions may alter the temporal variation of the confirmed cases. This change may affect the calibrating parameters of the mathematical prediction models. In other words, parameters of mathematical prediction models are required to be recalibrated when an effective intervention is applied. For this purpose, two scenarios were considered and compared for investigating the impact of applying preventive measurements to global health in Iran and Turkey. Since the daily number of confirmed and death cases dropped in April 2020 in Iran, the lockdown measures were relaxed, and the low-risk businesses were reopened on 18 April 2020 [20]. In this regard, two scenarios were considered to investigate the impact of this intervention for the COVID-19 outbreak in Iran: (1) a scenario without reopening the low-risk businesses on 18 April 2020 and (2) a scenario with reopening the low-risk businesses on 18 April 2020. The former scenario requires a new calibration, which is conducted in Figure 8(a), while the calibration presented in Figure 1(a) was used for the latter.  Figure 8(b) compares the total observed confirmed cases with the estimated ones based on the two scenarios considered. As shown, the estimated confirmed cases for the first and second scenarios are 92099 and 93888 cases on 2 May 2020, two weeks after reopening the low-risk businesses. Therefore, Figure 8(b) indicates that reopening the low-risk businesses increases the number of cumulative confirmed cases of COVID-19 up to more than 1780 cases in the next two weeks. This analysis indicates that even though the reopening the low-risk businesses was accompanied by social distancing and healthy protocols, it brought about an inevitable increase in positive cases in the next two weeks, which is confirmed with the observed confirmed cases in this period of time shown in Figure 8(b). With the increase of COVID-19 confirmed cases in Turkey, a total curfew was imposed on chronic patients and those whose ages are more than 65 years in late March. Also, mosques were closed on 16 March and several sports leagues were postponed on 19 March 2020 [21]. The impact of these preventive measurements was also investigated using two scenarios: (1) a scenario without intervention and (2) a scenario with intervention. The calibration process of the first scenario is shown in Figure 8(c), while Figure 1(b) presents the calibration process for the second scenario.  Figure 8(d) depicts the comparison of the observed confirmed cases and the two aforementioned scenarios. Based on Figure 8(d), applying preventive measurements reduced the accumulative number of positive cases of COVID-19 up to more than 24500 cases in two weeks after 19 March 2020. This considerable decrease is achieved by several preventive measurements like announcing curfew, closing mosques, and postponing sport events. This kind of analysis, which may provide a suitable perspective of the COVID-19 outbreak for health decision-makers, can be provided by applying mathematical prediction models.

The article "Assessment of Three Mathematical Prediction Models for Forecasting the COVID-19 Outbreak in Iran and Turkey" was published in 2020. Journal: Comput Math Methods Med.

The recursive-based prediction model requires the number of confirmed and death occurred at day *t* − 1 for prediction at day *t*, which may be one of the shortcomings of this prediction model. In other words, unlike the two other prediction models considered in this study, its input data is the confirmed and death of one day before, whereas the two other models work with the number of days passed from a certain time datum, which is mainly the first day that the first positive cases are identified. On the other hand, the recursive-based model needs two coefficients to be calibrated, while the Boltzmann function-based model and Beesham's model require the calibration of four and three coefficients, respectively. Thus, the fewer number of coefficients is one of the advantages of the recursive-based model in comparison with two other mathematical prediction models. Additionally, the structures of the recursive-based model and Beesham's model are much simpler for not only calibration but also application compared to that of the Boltzmann function-based model. Since applying preventive measurements may alter the outbreak trend, the calibration process of parameters of mathematical prediction models is commonly required to be repeated to take into account new changes. Although this may be counted as a drawback, it may provide an opportunity to investigate the impacts of applying preventive measurements by comparing the estimations of mathematical prediction models with or without such interventions. Such analysis may help to grasp an evidence-based perspective of the COVID-19 outbreak.

## 5. Conclusions

Although prediction of the COVID-19 pandemic may be inevitably accompanied by uncertainty, it may be useful for health politicians and public health decision-makers to plan and manage the outbreak of COVID-19. The recursive-based method, Boltzmann Function-based model, and Beesham's prediction model were used to forecast the COVID-19 outbreak from 20 February (for Iran) and 10 March 2020 (for Turkey) until 4 June 2020. The results indicate that the three models yielded to high values of determination coefficient, whereas their average absolute relative errors were significantly different. According to the comparison, the recursive-based model was found to be the most accurate prediction model, whereas the Boltzmann Function-based model estimated the COVID-19 outbreak with considerable average absolute relative errors. Furthermore, the former gave estimations with absolute relative errors lower than 0.1 for 75 (out of 85) and 51 (out of 65) days, while the corresponding values for the latter were 64 and 44 days for the confirmed cases of Iran and Turkey, respectively. Moreover, the recursive-based model estimated the closest peak confirmed cases to the observed data of Iran and Turkey, while the best predictions of the peak of death cases due to COVID-19 were obtained by the Boltzmann Function-based model. Additionally, the recursive-based model was employed to investigate the impacts of interventions. In this regard, it was found that reopening the low-risk businesses on 18 April 2020 in Iran increases the number of total positive cases up to more than 1780 cases during the next two weeks. Furthermore, conducting several control measurements in March 2020 was found to be effective in Turkey because it decreases the total number of COVID-19 confirmed cases up to more than 24500 cases in two weeks after 19 March 2020. Since the accuracy of prediction models of this pandemic plays a key role in adopting preventive measures, it is vital to exploit the one with the desirable precision.

The article "Assessment of Three Mathematical Prediction Models for Forecasting the COVID-19 Outbreak in Iran and Turkey" was published in 2020. Journal: Comput Math Methods Med.

## Figures and Tables

**Figure 1:** Recurrence plots for the confirmed and death cases of COVID-19 in Iran and Turkey.

**Figure 2:** Observed and estimated numbers of confirmed and death cases of COVID-19 in Iran and Turkey using the recursive-based model for the train data.

**Figure 3:** Observed and estimated numbers of confirmed and death cases of COVID-19 in Iran and Turkey using the Boltzmann function-based model for the train data.

**Figure 4:** Observed and estimated numbers of confirmed and death cases of COVID-19 in Iran and Turkey using Beesham's prediction model for the train data.

**Figure 5:** Comparison of the observed and estimated number of confirmed cases of COVID-19 for the test data using the recursive-based model in (a) Iran and (b) Turkey, using the recursive-based model in (c) Iran and (d) Turkey, and using Beesham's model in (e) Iran and (f) Turkey.

**Figure 6:** Comparison of the observed and estimated number of death cases of COVID-19 for the test data using the recursive-based model in (a) Iran and (b) Turkey, using the recursive-based model in (c) Iran and (d) Turkey, and using Beesham's model in (e) Iran and (f) Turkey.

**Figure 7:** Comparison of the three mathematical prediction models in terms of AARE for (a) confirmed cases of the train data, (b) confirmed cases of the test data, (c) death cases of the train data, and (d) death cases of the test data of the COVID-19 outbreak in Iran and Turkey.

The article "Assessment of Three Mathematical Prediction Models for Forecasting the COVID-19 Outbreak in Iran and Turkey" was published in 2020. Journal: Comput Math Methods Med.

**Figure 8:** Applying the recursive-based prediction model to different scenarios: (a) recurrence plots for the confirmed cases of Iran, (b) comparison of different scenarios for the confirmed cases of Iran, (c) recurrence plots for the confirmed cases of Turkey, and (d) comparison of different scenarios for the confirmed cases of Turkey.

**Table 1:** Comparison of the three mathematical models for estimating the peak values of confirmed and death cases of COVID-19 in Iran and Turkey.

Peak of the COVID-19 outbreak	Observed values	Estimated by the recursive-based model	Estimated by the Boltzmann function-based model	Estimated by Beesham's model
(a) Iran				
Confirmed cases (30 March 2020)	3186	2857	2302	1929
ARE	—	0.103	0.278	0.395
Death cases (5 April 2020)	158	134	156	108
ARE	—	0.152	0.015	0.314
(b) Turkey				
Confirmed cases (11 April 2020)	5138	4900	4225	3920
ARE	—	0.046	0.178	0.237
Death cases (19 April 2020)	127	117	130	105
ARE	—	0.079	0.021	0.170

## Data Availability

The data used in this study are available online (1, 14).
